The article "Edge Detection-Based Feature Extraction for the Systems of Activity Recognition" was published in 2022. Journal: Comput Intell Neurosci.

# Edge Detection-Based Feature Extraction for the Systems of Activity Recognition

**DOI:** 10.1155/2022/8222388

**Published:** 2022-01-31

**Authors:** Muhammad Hameed Siddiqi, Ibrahim Alrashdi

**Affiliations:** College of Computer and Information Sciences, Jouf University, Sakaka, Aljouf 2014, Saudi Arabia

## Abstract

Human activity recognition (HAR) is a fascinating and significant challenging task. Generally, the accuracy of HAR systems relies on the best features from the input frames. Mostly, the activity frames have the hostile noisy conditions that cannot be handled by most of the existing edge operators. In this paper, we have designed an adoptive feature extraction method based on edge detection for HAR systems. The proposed method calculates the direction of the edges under the presence of nonmaximum conquest. The benefits are in ease that depends upon the modest procedures, and the extension possibility is to determine other types of features. Normally, it is practical to extract extra low-level information in the form of features when determining the shapes and to get the appropriate information, the additional cultured shape detection procedure is utilized or discarded. Basically, this method enlarges the percentage of the product of the signal-to-noise ratio (SNR) and the highest isolation along with localization. During the processing of the frames, again some edges are demonstrated as a footstep function; the proposed approach might give better performance than other operators. The appropriate information is extracted to form feature vector, which further be fed to the classifier for activity recognition. We assess the performance of the proposed edge-based feature extraction method under the depth dataset having thirteen various kinds of actions in a comprehensive experimental setup.

## 1. Introduction

The extensive applications of human activity recognition (HAR) in real-time surveillance, athletics, human to human communication, and healthcare have illustrated significant effects in rearing the quality of human lives. In the domains of telemedicine and healthcare, the remote analysis of the patients' activities and well treatment might provide the innovation in the development of such domains. This type of development trains the physicians in their corresponding decision-making procedures through remotely watching the activities of the patients, specifically the stroke patients [1]. This process describes a case study for monitoring the critical situations of the stroke patients in telemedicine. The condition of the stroke patients might be explained through the methods of activity recognition systems, which might help the experts to provide the daily recommendations to the patients. The activities like jogging and walking might be recognized for the stroke patients, and hence the recommendations might be provided remotely for the better treatment. Similarly, the psychoanalyst may utilize the technology of telecare for treating a patient with upcoming-distressing anxiety illness (UDAI) by remotely watching the exercises [2]. The methods have been developed to watch heart condition of the patients through telecare [3], which is a major application for the actions analysis. These innovations enable the experts and doctors to professionally watch and manage the diseases of the patients.

The article "Edge Detection-Based Feature Extraction for the Systems of Activity Recognition" was published in 2022. Journal: Comput Intell Neurosci.

Generally, HAR systems are recognizing the corresponding actions performed by a human through the collected data from various resources. In HAR, activities based on 2D vision are affected by illumination, obstruction, and shadow in real-time domains [4]. Wearable sensor-based human activity recognition has significant accuracy and instantaneous performance [5]. However, the collection of human actions through accelerometers and gyroscopes decreases the ease of human body and terminates the spontaneity of human computer interaction [6]. Currently, in telemedicine and healthcare, domains such neutral knowledge along with video technologies are employed that rise concealment issues. Then, it might lead to conditions where the humans might not recognize that their isolated data has been propagated and consequently convert exposed to a risk [7]. Kinect depth camera only captures the depth data and does not expose the identity and other sensitive information of the human in healthcare domains. This characteristic makes the depth camera a best choice against RGB camera, and thus, we select the depth camera instead of utilizing RGB camera for the proposed methodology.

The recognition of human activities might be categorized in two categories: frame-based recognition and sequence-based recognition. In frame-based recognition, only the extant frame is utilized with or without the standard frame to identify the human activities from the inward video frames, while in sequence-based recognition, the regular motion of the feature points is considered amongst the current frame and the initial frame. Hence, the frame-based recognition might not have the capability accurately recognize the human activities; therefore, we focused on the sequence-based recognition in this work. Generally, the HAR systems have four stages: segmentation, feature extraction, feature selection, and recognition. A huge amount of work has been done for segmentation and recognition; however, very limited approaches have been proposed on feature extraction and selection. State-of-the-art methods are discussed in [8–10] for HAR system, where the authors proposed a new feature extraction method based on Haar wavelet transform to create the feature vector. Then, they utilized k-NN for recognizing the activities, and they claimed best accuracy. However, Haar wavelet transform has a technical limitation, which is not continuous and hence is not distinguishable [11]. Moreover, if the corresponding data is large, then the observation step of k-NN can be slow, which is one major limitation of k-NN. Similarly, activity recognition frameworks were developed by [12–14] that were based on temporal matching method in order to build the temporal features, which further define the difference of motion sequences from various time periods. However, most of these systems are too complex and inefficient for comprehensive dataset, due to which these systems dropped the classification rates.

The article "Edge Detection-Based Feature Extraction for the Systems of Activity Recognition" was published in 2022. Journal: Comput Intell Neurosci.

Hence, in this paper, we have designed an adoptive feature extraction method for HAR systems. The proposed method calculates the direction of the edges under the presence of nonmaximum conquest. The benefits are in ease that depends upon the modest procedures, and the extension possibility is to determine other types of features. Normally, it is practical to extract extra low-level information in the form of features when determining the shapes, and to get the appropriate information, the additional cultured shape detection procedure is utilized or discarded. As illustrated, the activity frames are very noisy, and before the analysis, it needs preprocessing; therefore, we used histogram equalization for this step. Moreover, the whole frames consist of features named sludge that may be noticed for various edge operators to extract the edge, though without considering noise. The feature vectors for the proposed methodology have been generated using hysteresis thresholding, where the thresholds were selected manually for the best performance. In the proposed methodology, the elementary factors nicely reply to the noise, and it is hard to choose a threshold which discloses a main portion of the sludge boundary. Basically, this method enlarges the percentage of the product of the signal-to-noise ratio (SNR) and the highest isolation along with localization. During the processing of the frames, again some edges are demonstrated as a footstep function; the proposed approach might give better performance than other operators. The appropriate information is extracted to form feature vector, which is further fed to the classifier for activity recognition. We assess the performance of the proposed edge-based feature extraction method under the depth dataset having thirteen various kinds of actions in a comprehensive experimental setup.

The article "Edge Detection-Based Feature Extraction for the Systems of Activity Recognition" was published in 2022. Journal: Comput Intell Neurosci.

The structure of the remaining paper is as follows. Some literature reviews are well described along with their shortcomings in Section 2. The proposed method is explained in Section 3, while the results along with some discussions are presented in Section 4. At the end, the conclusion of the paper is indicated in Section 5.

## 2. Related Work

Recently, activity recognition includes understanding of human movements against a succession of frame observations regarding ecological situations. The newly established commodity depth cameras dig out innovative potentials of dealing with such concern but provide some sole challenges as well. A state-of-the-art feature extraction method was designed by [15] for condensed system, which was based on spatial and temporal information. Further, they utilized k-NN for the classification, and they claimed higher performance accuracy. However, this system is complex and inefficient for comprehensive dataset, due to which this system dropped the classification rates, and that is one of the common limitations of spatial and temporal based features. Moreover, if the corresponding data is large, then the observation step of k-NN can be slow, which is one major limitation of k-NN [16]. Similarly, the authors of [17] developed a psychology-enthused twin stream gated recurring unit approach for activity classification that was based on human body joints. Their approach achieved an 89.97% classification accuracy. However, their approach might not be applicable in healthcare domains because of low accuracy.

A depth map-based HAR system was designed by [18, 19] that utilized convolutional autoencoder neural network in order to train and learn fixed features and summarize the gratified of single depth maps. However, convolutional neural network is not appropriate for naturalistic domains. Moreover, computational-wise, it is much expensive and needs special device for training [20]. Similarly, an ensembled method was developed by [21, 22] for HAR systems, which was based on graph network for human skeleton. The system utilized information fusion, deep learning, and temporal information in order to extract the best features. However, for data fusion, it is hard to establish applications and data in a precise level of the system and to reprocess it [23], also it is improper for human viewpoint [24]. Moreover, temporal-based information is inefficient for comprehensive dataset, due to which this system dropped the classification rates.

On the other hand, an integrated descriptor-based method was designed by [25] for HAR system. In this system, for feature extraction, the concept of multilevel fusion was utilized against depth frames to devise a comprehensive learning system. However, multilevel fusion-based feature extraction has some common issues like feature mismatch, robustness to camera sensors, letdown, and susceptibility to unpredictable noise or meddling because the distinction compassion greatly decreases the significant of multilevel fusion-based methods [26]. Furthermore, finding optimal features and feature extraction methods require extensive domain knowledge, which is time-consuming [27]. In the approach of [28], the authors improved the gesture, and still history frames are calculated, which further helped in the extraction of gradient feature [28]. However, one of the major limitations of gradient-based feature extraction technique is the existence of numerous local optima, resultant in explanations where global optimum might not simply be guaranteed [29].

The article "Edge Detection-Based Feature Extraction for the Systems of Activity Recognition" was published in 2022. Journal: Comput Intell Neurosci.

An efficient approach was proposed by [30] for HAR under three-dimensional skeleton information. In this approach, they simply employed a straight-forward deep learning model for activity classification. However, one of the major problems in skeleton-based feature extraction method is that the alone sparse skeleton data might not enough to completely classify the human activities [31]. Similarly, an improved bag-of-visual-words based activity classification method was designed by [32], where the authors employed support vector machine for classification. However, in this model, throughout the feature detection process, a huge number of key points are positioned that affect the performance of the model, due to which computational-wise, it is also more expensive [33]. Also, support vector machine is a vector-based classifier, which cannot classify the sequence-based activities. An adoptive state of the art approach was presented by [34] that was three-dimensional autocorrelation features. Moreover, they described the sequence of depth movement maps in order to get the data of temporal movement that might differentiate identical activities. However, this method is pretentious by affinal transformations that needs extra progresses to resolve 1 more complex activity recognition [35].

Therefore, the proposed method calculates the direction of the edges under the presence of nonmaximum conquest. The benefits are in ease that depends upon the modest procedures, and the extension possibility is to determine other types of features. Normally, it is practical to extract extra low-level information in the form of features when determining the shapes, and to get the appropriate information, the additional cultured shape detection procedure is utilized or discarded. Basically, this method enlarges the percentage of the product of the signal-to-noise ratio (SNR) and the highest isolation along with localization. During the processing of the frames, again some edges are demonstrated as a footstep function; the proposed approach might give better performance than other operators. The appropriate information is extracted to form feature vector, which is further fed to the classifier for activity recognition.

The article "Edge Detection-Based Feature Extraction for the Systems of Activity Recognition" was published in 2022. Journal: Comput Intell Neurosci.

## 3. Proposed Edge Detection Algorithm

The analysis of Taylor series tells that head-to-head pixel's differencing delivers the estimation of the first-order derivative at a pixel. If the variation is considered, then the pixels are divided by ∇*i*; then, by Taylor extension, *g*(*i*+∇*i*) is

(1) $$\begin{array}{c} g\left(i+\nabla i\right)=g\left(i\right)+\nabla i\times g^{\prime }\left(i\right)+\frac{\nabla i^{2}}{2!}\times g^{\prime \prime }\left(i\right)+Q\left(\nabla i^{3}\right). \end{array}$$

By reordering, the term *g*(*i*) is given as

(2) $$\begin{array}{c} g\left(i\right)=\frac{g\left(i+\nabla i\right)-g\left(i\right)}{\nabla i}-Q\left(\nabla i\right). \end{array}$$

These indicate the variations among the head-to-head pixels, that is, the estimation of the first order derivative along with error *Q*(∇*i*), which relies on the dimension of ∇*i* and the intricacy of the edge. If ∇*i* is high, then the error may be high. In training, the rapid selection of image points and the condensed high pitch content consider this assumption suitable, which is equal to calculating the difference of the first order that is carried out at two head-to-head pixels, which is a difference at horizontal such as *ε*_*d*_*xx*, which is given as follows:

(3) $$\begin{array}{c} \varepsilon_{d}xx_{i,j}=\varepsilon_{d}x_{i+1,j}+\varepsilon_{d}x_{i,j}\\ =\rho_{i+1,j}-\rho_{i,j}+\rho_{i,j}-\rho_{i-1,j}\\ =\rho_{i+1,j}-\rho_{i-1,j}, \end{array}$$

which is equal to integrating space to perceive the edges *ε*_*d*_*xx* by

(4) $$\begin{array}{c} \varepsilon_{d}xx_{i,j}=\left|=\rho_{i+1,j}-\rho_{i-1,j}\right|\forall i\in 2,\;K-1,\;j\in 1,K. \end{array}$$

Again, in order to analyze the Taylor series, we extend *g*(*i* − ∇*i*) as

(5) $$\begin{array}{c} g\left(i-\nabla i\right)=g\left(i\right)-\nabla i\times g^{\prime }\left(i\right)+\frac{\nabla i^{2}}{2!}\times g^{\prime \prime }\left(i\right)-Q\left(\nabla i^{3}\right). \end{array}$$

By substituting equations (1) and (5), we achieve the following:

(6) $$\begin{array}{c} g^{\prime }\left(i\right)=\frac{g\left(i+\nabla i\right)-g\left(i-\nabla i\right)}{2\nabla i}-Q\left(\nabla i^{2}\right). \end{array}$$

Equation (6) recommends that currently, the estimation of the first order variation is the variation among the pixels detached by a single point along with *Q*(∇*i*^2^). If ∇*i* < 1, which is obviously lesser than the integrated error of head-to-head pixels (as shown in equation (6)), which further can be utilized by noise or error reduction as

(7) $$\begin{array}{c} \varepsilon_{d_{i,j}}=\max\left\{\left|M^{+}*\rho_{i,j}\right|,\left|M^{-}*\rho_{i,j}\right|\right\}\;\forall i,j\in 1,\;K-1. \end{array}$$

*M* is the length between the edge direction and vector. During implementation, those templates which provided the highest value are stored as the edge value at that pixel. Then, the pixel of the edge *ε*_*d*_*i*,*j*__ is the highest for two values originated through the convolution of the two image templates at point *ρ*_*i*,*j*_.

The article "Edge Detection-Based Feature Extraction for the Systems of Activity Recognition" was published in 2022. Journal: Comput Intell Neurosci.

Another way of considering the highest value is only the summation of results of the two templates to associate the edges along horizontal and vertical. There are various diversities of the edges that mostly be utilized to take the two templates as one of the facilitating mechanisms to build an *edge vector* along horizontal axis and vertical axis, respectively. Edge detection is a kind of mechanism to differentiate the two things, as it perceives variations, which must reply to noise and step-like image intensity variations in image intensity. Therefore, it is practical to integrate the average in the process of edge detection. Hence, we may spread the horizontal (*M*_*i*_) and vertical (*M*_*j*_) templates along three rows and columns, respectively, which provides two types of results such as the brightness on every axis and magnitude of the edge; *θ* is the vector angle, which is explained as follows:

(8) $$\begin{array}{c} M\left(i,j\right)=\sqrt{M_{i}{\left(i,j\right)}^{2}+M_{j}{\left(i,j\right)}^{2}},\\ \vartheta \left(i,j\right)={\text{tan}}^{-1}\left(\frac{M_{i}\left(i,j\right)}{M_{j}\left(i,j\right)}\right). \end{array}$$

*M*_*i*_ and *M*_*j*_ might be utilized to find the suitable quadrangle for the direction of the edge. In the proposed methodology, we also utilized Sobel operator, which employs two windows in order to find the edges in the form of vectors, and it is one of the most well-known edge detection operators. Moreover, the proposed method along with Sobel operator showed better performance against other concurrent operators. The proposed operator also considers the optimum averaging procedures and differencing. The Gaussian averaging has previously quantified to provide the optimum averaging. The binomial theorem provides a series of integer coefficients in order to approximate the normal distribution. As described before, we are utilizing two windows that provide us two sets of coefficients in the form of triangles as shown in Figure 1.

The article "Edge Detection-Based Feature Extraction for the Systems of Activity Recognition" was published in 2022. Journal: Comput Intell Neurosci.

Figure 1(a) provides the irregular coefficients of an optimum discrete sharpening operator, which is basically a Gaussian filter along with integer coefficients. In Figure 1, the increasing coefficients for the window is given by the rows. The coefficients of sharpening inside the Sobel operator are of size 3 × 3. Moreover, Figure 1(b) describes the Pascal triangle coefficients for the subtraction, which might be executed by deducting the templates derived from the corresponding head-to-head extensions for the size of minor mask. Therefore, we need a filter that might offer the Pascal triangle coefficients for window parameters such that size is *p* and location is *γ*. The filter is the Pascal (*γ*, *p*) as shown in the following:

(9) $$\begin{array}{c} \text{Pascal}\left(\gamma ,p\right)=\left|\begin{array}{cc} \frac{p!}{\left(p-\gamma \right)!*\gamma !} & \text{if }\left(0\leq \gamma \leq p\right)\\ 0 & \text{otherwise} \end{array}\right|. \end{array}$$

There are four possibilities for the edge direction measurement delivered by the Sobel operator, as described in Figure 2.

In Figure 2, the reversing template of *M*_*i*_ does not specify the disjointedness at the turnings, which means the magnitude of the edge under the presence of the Sobel employed to the square is not presented but is comparable to those operators originated by the applications of other operators. If we change the templates of the Sobel filter, the edges' direction measurement is organized and may be the normal edges by itself. But when the edges are to be determined, the reorganization might help in the construction of the algorithm to find the target. So, for this purpose, if an algorithm is locating the shapes, then it must use the direction of the edges for the accurate preparation. This procedure might improve the performance of the algorithm, but it must precisely map the corresponding image data. Once all the edges and their corresponding directions are detected, then the entire information has been stored in the form of feature vector, which is further utilized in hidden Markov model for activity recognition.

## 4. Algorithm Evaluation

We evaluated the proposed methodology against the following flow.

### 4.1. Arrangement for Experiments

We performed the following experiments in order to judge the performance of the proposed methodology:

- The first experiment indicates the accuracy of the proposed methodology against the defined dataset. An *n* – 1-fold cross justification scheme has been used for the entire experiments, which means that the data from each subject will be utilized at least once for training and testing in order to maintain the robustness.
- In the second experiment, comprehensive experiments are presented instead of using the proposed methodology, which means that we will perform multiple experiments with recent feature extraction methods but will not utilize the proposed feature extraction method.
- In the final experiment, state-of-the-art methods are compared with the performance of the proposed methodology.

The article "Edge Detection-Based Feature Extraction for the Systems of Activity Recognition" was published in 2022. Journal: Comput Intell Neurosci.

### 4.2. Depth Images Dataset

This defined dataset has a sequence of 670 videos, which were collected under the setting of Kinect depth camera. There were a total 70 subjects (university students: male and female) that performed thirteen activities such as bending, jacking, place-jumping, running, side movement, skipping, walking, one-hand waving, two-hand waving, jumping, clapping, boxing, and sitting up and down. In order to make the dataset more realistic, we recorded some videos from stroke patients in real healthcare domain. All the activity frames have various sizes; therefore, we have reduced the sizes of the entire frames to 100 × 100 in order to sustain the normalization. The dataset was recorded in 6-month period (from February 2017 to July 2017).

### 4.3. Experimental Results and Discussions

In the first experiment, we presented the accuracy of the proposed methodology against the depth dataset, which are performed in MATLAB using offline setting in lab. The whole results are represented in Table 1.

The proposed methodology showed significant accuracy, as presented in Table 1. This significant performance is of the calculation of the edge directions under the presence of nonmaximum conquest. Also, during the processing of the frames, some edges are demonstrated as a footstep function; the proposed approach might give better performance than other operators.

In the second experiment, the accuracies are represented against various latest feature extraction methods of machine learning. However, in these experiments, we will not use the proposed methodology. For these group of experiments, we employed different types of well-known feature extraction techniques such as autoencoder, histogram of oriented gradients, contrast features, ellipse features, Fourier features, Gabor features, Haralick texture features, geometric features, local binary pattern features, and basic intensity features. The whole results for this group of experiments against depth dataset are described in Tables 2–11, respectively.

As demonstrated in Tables 2–11, the proposed activity recognition system did not get best classification rates with latest feature extraction techniques. On the other side, the system achieved significant accuracy with the proposed feature extraction technique. This is because the proposed method calculates the direction of the edges under the presence of nonmaximum conquest. The benefits are in ease that depends upon the modest procedures, and the extension possibility is to determine other types of features. Normally, it is practical to extract extra low-level information in the form of features when determining the shapes, and to get the appropriate information, the additional cultured shape detection procedure is utilized or discarded.

The article "Edge Detection-Based Feature Extraction for the Systems of Activity Recognition" was published in 2022. Journal: Comput Intell Neurosci.

In the last experiment, the accuracy of classification for the proposed methodology is compared with the state of the art HAR systems. In the existing systems, some of the systems are executed for these experiments, while for some systems, we borrowed their simulation, and for some systems, we took the results from their corresponding papers. All of the systems are implemented against the depth dataset with the exact sceneries as presented in their respective works. The whole comparison results are indicated in Table 12.

As demonstrated in Table 12, the proposed methodology achieved the highest accuracy on depth dataset compared to other state-of-the-art systems. This is because in the proposed method, during the processing of the frames, some edges are demonstrated as a footstep function; the proposed approach might give better performance than other operators. Also, some appropriate information is extracted to form feature vector, which is further fed to the classifier to get best accuracy of classification.

## 5. Conclusion

Human activity recognition states the task of evaluating the physical activity of a person over the usage of neutral knowledge. Currently, in telemedicine and healthcare domains, such neutral knowledge, along with video technologies, is employed, which rise concealment issues; then, it might lead to conditions where the humans might not recognize that their isolated data has been propagated and consequently convert exposed to a risk. Therefore, in this paper, we have designed an adoptive feature extraction method for HAR systems, which utilized Kinect depth camera in order to resolve the privacy issue. The proposed method calculates the direction of the edges under the presence of nonmaximum conquest. The benefits are in ease that depends upon the modest procedures, and the extension possibility is to determine other types of features. Normally, it is practical to extract extra low-level information in the form of features when determining the shapes, and to get the appropriate information, the additional cultured shape detection procedure is utilized or discarded. The benefits are in ease that depends upon the modest procedures, and the extension possibility is to determine other types of features. Normally, it is practical to extract extra low-level information in the form of features when determining the shapes, and to get the appropriate information, the additional cultured shape detection procedure is utilized or discarded. As illustrated, the activity frames are very noisy, and before the analysis, it needs preprocessing; therefore, we used histogram equalization for this step. Moreover, the whole frames consist of features named sludge that may be noticed for various edge operators to extract the edge, though without considering noise. The feature vectors for the proposed methodology have been generated using hysteresis thresholding, where the thresholds were selected manually for the best performance. In the proposed methodology, the elementary factors nicely reply to the noise, and it is hard to choose a threshold which discloses a main portion of the sludge boundary. Basically, this method enlarges the percentage of the product of the signal-to-noise ratio (SNR) and the highest isolation along with localization. During the processing of the frames, again some edges are demonstrated as a footstep function; the proposed approach might give better performance than other operators. The appropriate information is extracted to form feature vector, which is further fed to the classifier for activity recognition. We assess the performance of the proposed edge-based feature extraction method under the depth dataset having thirteen various kinds of actions in a comprehensive experimental setup. The proposed methodology achieved the highest accuracy of classification compared to the existing latest HAR systems.

The article "Edge Detection-Based Feature Extraction for the Systems of Activity Recognition" was published in 2022. Journal: Comput Intell Neurosci.

In the future, we will try to improve the proposed methodology in the telemedicine and healthcare domains in order to sustain the same accuracy and facilitate the physicians for better recommendations. Moreover, our alternative goal is to deploy the proposed methodology in smart phones. So, for that purpose, we will try to propose a light weight classifier coupled with the proposed approach to implement it in the smart phone for real healthcare domains.

## Figures and Tables

**Figure 1:** (a) The additive Pascal triangle and (b) the subtractive Pascal triangle for the set of coefficients.

**Figure 2:** Another preparation of edge direction. (a) (*M*_*i*_, *M*_*j*_), (b) (−*M*_*i*_, *M*_*j*_), (c) (*M*_*j*_, *M*_*i*_), and (d) (−*M*_*j*_, −*M*_*i*_), respectively.

**Table 1:** Accuracy of classification for the proposed methodology against depth dataset.

Activities	BN	JC	PLJ	RNN	SIM	SKP	WLK	OW1	OW2	JP	CLP	BXG	SUD
BN	**98**	0	0	0	0	2	0	0	0	0	0	0	0
JC	0	**97**	1	0	0	2	0	0	0	0	0	0	0
PLJ	0	0	**99**	0	0	0	0	1	0	0	0	0	0
RNN	0	2	0	**96**	0	0	1	0	0	1	0	0	0
SIM	0	0	0	0	**100**	0	0	0	0	0	0	0	0
SKP	0	0	1	0	0	**95**	1	0	1	0	1	0	1
WLK	0	0	0	0	0	0	**100**	0	0	0	0	0	0
OW1	0	0	0	0	1	0	0	**99**	0	0	0	0	0
OW2	1	0	0	0	0	1	0	0	**97**	0	0	1	0
JP	0	0	1	0	0	0	0	1	0	**98**	0	0	0
CLP	0	0	0	0	0	1	0	0	0	0	**99**	0	0
BXG	0	2	0	1	0	0	1	0	0	0	0	**96**	0
SUD	0	0	0	0	1	0	0	0	0	0	0	0	**99**

Average	**97.9%**												

BN for bending, JC for jacking, PLJ for place jumping, RNN for running, SIM for side movement, SKP for skipping, WLK for walking, OW1 for one-hand waving, OW2 for two-hand waving, JP for jumping, CLP for clapping, BXG for boxing, and SUD for sitting up and down

**Table 2:** Accuracy of classification for the proposed activity recognition system with autoencoder (without employing the proposed methodology) against depth dataset.

Activities	BN	JC	PLJ	RNN	SIM	SKP	WLK	OW1	OW2	JP	CLP	BXG	SUD
BN	**80**	0	2	3	1	2	0	5	1	0	2	4	0
JC	1	**79**	1	3	1	2	2	4	2	1	0	3	1
PLJ	0	2	**84**	1	0	3	0	2	0	4	0	2	2
RNN	4	2	1	**77**	3	1	1	6	2	1	0	1	1
SIM	2	1	2	4	**79**	1	2	1	3	0	2	1	2
SKP	2	2	1	2	1	**81**	1	3	1	0	3	2	1
WLK	0	2	3	0	1	2	**85**	2	1	1	2	0	1
OW1	3	1	2	2	4	2	2	**75**	2	2	1	3	1
OW2	1	0	2	1	2	2	1	3	**80**	1	2	1	4
JP	2	1	1	2	3	2	1	1	2	**82**	2	1	1
CLP	2	3	0	1	1	1	2	0	4	2	**83**	1	0
BXG	2	2	1	1	2	4	1	2	1	1	2	**79**	2
SUD	0	1	4	2	1	0	2	1	0	2	1	0	**86**

Average	**81.5%**												

BN for bending, JC for jacking, PLJ for place jumping, RNN for running, SIM for side movement, SKP for skipping, WLK for walking, OW1 for one-hand waving, OW2 for two-hand waving, JP for jumping, CLP for clapping, BXG for boxing, and SUD for sitting up and down.

**Table 3:** Accuracy of classification for the proposed activity recognition system with histogram of oriented gradients (without employing the proposed methodology) against depth dataset.

Activities	BN	JC	PLJ	RNN	SIM	SKP	WLK	OW1	OW2	JP	CLP	BXG	SUD
BN	**83**	0	2	1	2	2	0	3	1	0	2	1	3
JC	0	**87**	1	2	0	2	1	2	0	2	0	2	1
PLJ	2	2	**80**	2	1	2	2	1	2	1	2	2	1
RNN	3	2	2	**79**	3	1	4	0	2	1	2	1	0
SIM	1	3	1	2	**82**	2	2	2	1	2	1	0	1
SKP	0	2	1	3	2	**85**	1	2	1	0	1	1	1
WLK	2	2	0	1	4	2	**78**	1	4	1	2	2	1
OW1	0	5	2	2	1	3	3	**76**	2	3	1	2	0
OW2	3	2	1	2	2	1	5	2	**72**	1	5	2	2
JP	2	2	4	1	2	2	1	1	3	**76**	1	1	4
CLP	1	0	1	2	1	1	2	4	1	2	**80**	2	3
BXG	0	1	2	1	1	3	2	1	2	2	1	**82**	2
SUD	1	2	1	0	1	0	3	1	2	1	3	2	**83**

Average	**80.2%**												

BN for bending, JC for jacking, PLJ for place jumping, RNN for running, SIM for side movement, SKP for skipping, WLK for walking, OW1 for one-hand waving, OW2 for two-hand waving, JP for jumping, CLP for clapping, BXG for boxing, and SUD for sitting up and down.

The article "Edge Detection-Based Feature Extraction for the Systems of Activity Recognition" was published in 2022. Journal: Comput Intell Neurosci.

**Table 4:** Accuracy of classification for the proposed activity recognition system with contrast features (without employing the proposed methodology) against depth dataset.

Activities	BN	JC	PLJ	RNN	SIM	SKP	WLK	OW1	OW2	JP	CLP	BXG	SUD
BN	**88**	0	2	2	1	2	1	1	0	2	0	1	0
JC	0	**89**	1	1	2	2	0	2	1	0	1	0	1
PLJ	2	0	**90**	2	1	0	1	1	0	2	0	1	0
RNN	1	2	1	**85**	0	2	1	2	2	1	1	0	2
SIM	0	1	2	2	**87**	1	2	0	2	1	0	2	0
SKP	2	1	1	1	2	**83**	1	2	1	2	1	2	1
WLK	1	2	2	2	1	2	**80**	1	2	1	3	1	2
OW1	4	1	2	1	1	2	2	**78**	1	2	1	2	3
OW2	1	2	5	2	3	1	2	2	**77**	1	2	1	1
JP	2	2	1	0	1	2	2	1	2	**82**	2	2	1
CLP	1	1	2	2	1	1	3	2	1	0	**81**	4	1
BXG	2	2	3	1	2	1	1	2	1	1	2	**80**	2
SUD	0	1	1	2	1	1	2	1	2	1	2	0	**86**

Average	**83.5%**												

BN for bending, JC for jacking, PLJ for place jumping, RNN for running, SIM for side movement, SKP for skipping, WLK for walking, OW1 for one-hand waving, OW2 for two-hand waving, JP for jumping, CLP for clapping, BXG for boxing, and SUD for sitting up and down.

**Table 5:** Accuracy of classification for the proposed activity recognition system with ellipse features (without employing the proposed methodology) against depth dataset.

Activities	BN	JC	PLJ	RNN	SIM	SKP	WLK	OW1	OW2	JP	CLP	BXG	SUD
BN	**90**	0	2	1	0	2	1	0	1	0	1	0	2
JC	0	**91**	1	0	0	2	1	0	2	2	0	1	0
PLJ	2	0	**88**	1	2	0	0	1	2	0	1	2	1
RNN	0	2	2	**86**	0	1	1	2	0	1	3	0	2
SIM	2	1	1	2	**80**	2	1	1	2	2	1	2	3
SKP	1	2	1	0	2	**83**	1	4	1	0	2	2	1
WLK	0	1	0	2	0	2	**91**	0	1	1	2	0	0
OW1	2	0	2	1	1	2	1	**84**	2	2	0	1	2
OW2	1	2	1	2	1	1	0	2	**86**	0	2	1	1
JP	2	1	1	0	2	0	1	1	0	**89**	1	2	0
CLP	1	0	1	0	2	1	0	1	0	1	**92**	0	1
BXG	1	2	1	1	0	2	1	0	2	0	1	**89**	0
SUD	0	1	0	2	1	0	2	0	1	1	0	2	**90**

Average	**87.6%**												

BN for bending, JC for jacking, PLJ for place jumping, RNN for running, SIM for side movement, SKP for skipping, WLK for walking, OW1 for one-hand waving, OW2 for two-hand waving, JP for jumping, CLP for clapping, BXG for boxing, and SUD for sitting up and down.

**Table 6:** Accuracy of classification for the proposed activity recognition system with Fourier features (without employing the proposed methodology) against depth dataset.

Activities	BN	JC	PLJ	RNN	SIM	SKP	WLK	OW1	OW2	JP	CLP	BXG	SUD
BN	**93**	0	2	1	0	2	0	1	0	1	0	0	0
JC	1	**89**	1	0	1	2	1	0	2	0	2	0	1
PLJ	0	2	**91**	1	0	1	0	1	1	0	1	2	0
RNN	0	0	0	**94**	1	0	1	0	0	1	0	1	2
SIM	2	1	1	0	**87**	2	1	1	2	0	2	0	1
SKP	4	0	1	2	2	**83**	1	0	1	2	1	2	1
WLK	0	2	0	1	0	2	**90**	1	0	2	0	2	0
OW1	1	0	2	1	2	0	2	**87**	1	0	2	0	2
OW2	1	2	0	2	1	1	0	2	**88**	1	1	1	0
JP	0	1	1	0	2	0	2	1	0	**91**	0	2	0
CLP	1	0	2	1	0	1	0	1	1	0	**92**	0	1
BXG	1	2	0	1	2	0	1	0	0	2	0	**89**	2
SUD	2	1	2	0	1	2	2	1	2	1	1	2	**83**

Average	**89.0%**												

BN for bending, JC for jacking, PLJ for place jumping, RNN for running, SIM for side movement, SKP for skipping, WLK for walking, OW1 for one-hand waving, OW2 for two-hand waving, JP for jumping, CLP for clapping, BXG for boxing, and SUD for sitting up and down.

The article "Edge Detection-Based Feature Extraction for the Systems of Activity Recognition" was published in 2022. Journal: Comput Intell Neurosci.

**Table 7:** Accuracy of classification for the proposed activity recognition system with Gabor features (without employing the proposed methodology) against depth dataset.

Activities	BN	JC	PLJ	RNN	SIM	SKP	WLK	OW1	OW2	JP	CLP	BXG	SUD
BN	**91**	2	0	1	0	2	0	0	1	0	1	2	0
JC	0	**90**	1	2	0	2	0	2	0	1	0	1	1
PLJ	2	0	**86**	1	2	0	2	1	1	0	2	1	2
RNN	1	2	1	**84**	1	2	1	0	2	1	1	2	2
SIM	0	1	0	1	**92**	0	2	1	0	2	1	0	0
SKP	1	0	1	1	0	**93**	1	0	1	0	1	0	1
WLK	2	1	0	2	1	0	**89**	2	0	1	0	2	0
OW1	2	0	1	0	1	0	2	**88**	0	2	0	2	2
OW2	1	2	0	1	0	1	0	0	**94**	0	0	1	0
JP	0	1	1	0	2	0	2	1	1	**87**	2	1	2
CLP	2	0	2	1	0	1	1	2	2	1	**85**	2	1
BXG	1	2	0	1	2	0	1	0	1	0	1	**91**	0
SUD	2	0	1	0	1	1	0	2	1	1	0	1	**90**

Average	**89.2%**												

BN for bending, JC for jacking, PLJ for place jumping, RNN for running, SIM for side movement, SKP for skipping, WLK for walking, OW1 for one-hand waving, OW2 for two-hand waving, JP for jumping, CLP for clapping, BXG for boxing, and SUD for sitting up and down.

**Table 8:** Accuracy of classification for the proposed activity recognition system with Haralick texture features (without employing the proposed methodology) against depth dataset.

Activities	BN	JC	PLJ	RNN	SIM	SKP	WLK	OW1	OW2	JP	CLP	BXG	SUD
BN	**88**	0	2	1	1	2	0	1	2	1	0	2	0
JC	1	**90**	1	2	0	2	1	0	1	0	1	0	1
PLJ	0	2	**85**	0	2	0	2	1	2	1	1	2	2
RNN	2	2	1	**79**	1	2	1	2	1	1	4	2	2
SIM	1	3	2	1	**77**	4	2	1	3	2	1	2	1
SKP	2	1	1	2	2	**81**	1	2	1	2	1	3	1
WLK	1	2	2	1	0	1	**83**	1	2	1	2	1	2
OW1	2	1	2	2	1	2	1	**76**	2	2	1	2	6
OW2	1	2	1	1	2	1	0	2	**86**	1	2	0	1
JP	0	1	1	2	0	0	2	1	0	**92**	0	1	0
CLP	2	0	2	0	2	1	1	0	1	2	**87**	0	2
BXG	1	2	0	1	1	0	1	2	0	1	1	**89**	1
SUD	0	1	2	0	1	1	0	0	1	0	2	1	**91**

Average	**84.9%**												

BN for bending, JC for jacking, PLJ for place-jumping, RNN for running, SIM for side movement, SKP for skipping, WLK for walking, OW1 for one-hand waving, OW2 for two-hand waving, JP for jumping, CLP for clapping, BXG for boxing, and SUD for sitting up and down.

**Table 9:** Accuracy of classification for the proposed activity recognition system with geometric features (without employing the proposed methodology) against depth dataset.

Activities	BN	JC	PLJ	RNN	SIM	SKP	WLK	OW1	OW2	JP	CLP	BXG	SUD
BN	**79**	2	3	1	2	2	1	4	2	1	1	0	2
JC	2	**77**	1	2	5	2	2	1	3	2	2	1	0
PLJ	1	2	**83**	2	2	1	2	1	1	2	0	2	1
RNN	0	2	1	**86**	1	2	1	2	0	1	2	0	2
SIM	2	1	0	2	**90**	0	1	1	0	2	0	1	0
SKP	0	2	1	0	2	**88**	0	2	1	0	1	2	1
WLK	2	1	2	1	1	2	**81**	1	2	2	2	1	2
OW1	1	1	1	2	1	1	2	**84**	1	2	1	2	1
OW2	1	0	2	1	2	1	0	2	**87**	1	2	1	0
JP	2	1	1	2	1	2	2	1	2	**78**	2	2	4
CLP	2	5	2	1	2	1	3	2	1	2	**75**	3	1
BXG	1	1	0	1	2	2	1	0	1	1	1	**89**	0
SUD	0	2	1	0	1	0	0	1	0	2	0	2	**91**

Average	**83.7%**												

BN for bending, JC for jacking, PLJ for place jumping, RNN for running, SIM for side movement, SKP for skipping, WLK for walking, OW1 for one-hand waving, OW2 for two-hand waving, JP for jumping, CLP for clapping, BXG for boxing, and SUD for sitting up and down.

The article "Edge Detection-Based Feature Extraction for the Systems of Activity Recognition" was published in 2022. Journal: Comput Intell Neurosci.

**Table 10:** Accuracy of classification for the proposed activity recognition system with local binary pattern features (without employing the proposed methodology) against depth dataset.

Activities	BN	JC	PLJ	RNN	SIM	SKP	WLK	OW1	OW2	JP	CLP	BXG	SUD
BN	**93**	0	0	1	0	2	0	1	0	0	2	0	1
JC	0	**91**	1	0	1	2	0	0	2	1	0	2	0
PLJ	2	0	**89**	2	1	0	2	1	0	0	1	0	2
RNN	1	2	0	**86**	2	1	1	2	1	1	0	2	1
SIM	1	0	2	0	**92**	2	0	1	0	0	1	1	0
SKP	2	1	1	1	0	**89**	1	0	1	2	1	0	1
WLK	0	2	0	0	2	0	**94**	0	0	0	0	2	0
OW1	2	0	1	2	1	1	0	**84**	2	1	2	2	2
OW2	1	2	2	1	2	1	1	2	**80**	2	1	1	4
JP	1	1	1	2	2	2	1	1	0	**82**	2	3	2
CLP	0	2	1	1	0	1	2	2	2	0	**88**	1	0
BXG	1	2	0	1	1	0	1	0	0	2	0	**91**	1
SUD	2	0	2	1	1	2	0	2	2	0	2	0	**86**

Average	**88.0%**												

BN for bending, JC for jacking, PLJ for place jumping, RNN for running, SIM for side movement, SKP for skipping, WLK for walking, OW1 for one-hand waving, OW2 for two-hand waving, JP for jumping, CLP for clapping, BXG for boxing, and SUD for sitting up and down.

**Table 11:** Accuracy of classification for the proposed activity recognition system with basic intensity features (without employing the proposed methodology) against depth dataset.

Activities	BN	JC	PLJ	RNN	SIM	SKP	WLK	OW1	OW2	JP	CLP	BXG	SUD
BN	**79**	2	1	4	2	2	1	2	1	2	2	1	1
JC	1	**81**	1	2	1	2	2	1	2	1	2	2	2
PLJ	0	2	**84**	0	2	1	2	1	1	2	2	1	2
RNN	2	2	1	**76**	6	1	1	3	2	1	1	2	2
SIM	1	0	2	2	**90**	1	0	0	1	2	0	1	0
SKP	2	2	1	4	2	**74**	2	3	2	2	1	4	1
WLK	2	4	2	1	2	5	**73**	2	3	1	2	1	2
OW1	1	1	2	2	1	2	4	**78**	1	4	1	2	1
OW2	1	2	1	1	2	1	1	2	**85**	1	2	1	0
JP	2	1	2	2	1	2	0	1	2	**82**	1	2	2
CLP	2	1	2	2	2	1	1	1	2	2	**80**	2	2
BXG	1	2	4	1	2	2	1	2	1	2	4	**77**	1
SUD	2	6	1	2	1	1	2	4	2	1	2	4	**72**

Average	**79.3%**												

BN for bending, JC for jacking, PLJ for place jumping, RNN for running, SIM for side movement, SKP for skipping, WLK for walking, OW1 for one-hand waving, OW2 for two-hand waving, JP for jumping, CLP for clapping, BXG for boxing, and SUD for sitting up and down.

**Table 12:** Accuracies of classification for the proposed methodology along with the recent human activity recognition systems.

Recent systems	Accuracies of classification (%)	Std. dev. (*σ*)
[36]	89.2	±3.8
[37]	93.1	±1.3
[38]	85.9	±4.5
[39]	90.7	±3.6
[40]	81.6	±2.9
[41]	79.8	±1.6
[42]	88.5	±4.8

Proposed methodology	**97.9**	±2.1

The article "Edge Detection-Based Feature Extraction for the Systems of Activity Recognition" was published in 2022. Journal: Comput Intell Neurosci.

## Data Availability

The data used for this study and simulation will be provided on demand.
